# Clinical Performance Study of a New Fully Automated Red Blood Cell Permeability Fragility Analyzer

**DOI:** 10.1155/2022/5642907

**Published:** 2022-03-29

**Authors:** Shiwen Zheng, Qiuyan Li, Tong Ou, Yuqing Li, Song Wu

**Affiliations:** ^1^Medical College, Anhui University of Science and Technology, Huainan 232000, China; ^2^Shenzhen Following Precision Medical Research Institute, The Third Affiliated Hospital of Shenzhen University (Luohu Hospital Group), Shenzhen 518001, China; ^3^Shengli Clinical Medical College of Fujian Medical University and Department of Urology, Fujian Provincial Hospital, Fuzhou 350001, China

## Abstract

In order to verify the applicability of the erythrocyte fragility test (EFT) carried out by the new fully automatic erythrocyte permeability fragility analyzer RA-800 for thalassemia screening, a total of 100 cases of suspected thalassemia patients who underwent pregnancy examinations at Luohu District People's Hospital are included. The results of a new automatic erythrocyte permeability fragility analyzer RA-800 are compared with the results of the detection system composing of the KOFA erythrocyte fragility test kit currently used in clinical laboratories. The diagnosis confirmed by genetic testing is used as the gold standard to evaluate the applicability of RA-800. The sensitivity, specificity, and accuracy of the new automatic erythrocyte permeability fragility analyzer RA-800 screening for thalassemia were 66.67%, 92.86%, and 85.00%. The KOFA direct colorimetries are 76.67%, 81.43%, and 80.00%. The kappa value for the screening of thalassemia was 0.558, which concludes that the consistency was moderate. The ROC curve indicates that both two methods had diagnostic significance for the diagnostic value of thalassemia. The new automatic erythrocyte permeability fragility analyzer RA-800 is suitable for thalassemia screening, and the performance indexes meet the clinical requirements.

## 1. Introduction

Thalassemia is a group of genetic diseases caused by the reduction of hemoglobin *α* or *β*-chain synthesis [1]. It is one of the most common single-gene genetic diseases in humans. It is manifested as an imbalance in the ratio of *α*/*β*-globin chains leading to ineffective erythropoiesis, insufficient erythropoiesis, chronic hemolytic anemia, compensatory hematopoietic expansion, hypercoagulability, and increased intestinal iron absorption [2]. The disease is widely distributed around the world. The prevention of thalassemia can reduce birth defects and is of great significance to improving the quality of the population [3–5]. The clinical phenotypes of thalassemia gene carriers are highly heterogeneous, so genetic diagnosis is the gold standard for the diagnosis of thalassemia [6, 7]. Genetic testing can accurately diagnose thalassemia, but the testing is cumbersome, costly, and time-consuming, resulting in a waste of medical resources [8, 9]. It is difficult to promote in primary hospitals, communities, and areas with underdeveloped economies. Therefore, simple and economical screening indicators such as blood routine parameters, EFT, and Hb electrophoresis still play an indispensable role. At present, EFT detection kits are mostly used in clinics to use automatic biochemical analyzers for detection, and there are few instruments that specifically detect EFT [10].

The new automatic erythrocyte permeability fragility analyzer RA-800 used in this study uses the scattering turbidimetry to determine the erythrocyte permeability fragility. RA-800 has the advantages of simple operation, low cost, samples directly on the machine without any pretreatment, and no need to establish a laboratory assembly line. It is a single machine that can complete the measurement and fully realize the advantages of lightweight automated analysis. In this study, we will study the applicability of its clinical detection EFT for reference by the majority of clinical laboratory personnel and doctors.

## 2. Materials and Methods

### 2.1. Patients

From January 2021 to December 2021, a total of 100 cases of suspected thalassemia patients who underwent pregnancy examination and physical examination at Luohu District People's Hospital were the subjects of the study. A comparative study of the clinical performance test was carried out on the new automatic red blood cell permeability fragility analyzer RA-800, and the genetic test results were used as the gold standard.

### 2.2. Instruments and Methods

#### 2.2.1. Erythrocyte Permeability Fragility Test

RA-800: after anticoagulant whole blood is mixed, it is directly measured by RA-800 using scattering turbidimetry. The detection value is based on the hemolysis percentage less than 65% as the cutoff value.

KOFA: after anticoagulated whole blood is mixed, 20 *μ*L of whole blood cells is drawn and added to 1 mL of the sample treatment solution of the KOFA kit. After fully mixing, it is measured by the Beckman AU680 biochemical analyzer with direct colorimetry. The detection value is based on the cutoff value of hemolysis percentage less than 68%.

#### 2.2.2. Thalassemia Gene Test

After the peripheral blood DNA was extracted, there were three deletion types of *α*-thalassemia gene mutation types (--^SEA^, −*α*^3.7^, and −*α*^4.2^), three common nondeletion types of *α*-thalassemia gene mutation types (*α*^cs^, *α*^qs^, and *α*^ws^), and seventeen common mutation types of *β*-thalassemia genes will be tested using the thalassemia gene kit. The experimental process was carried out by the members of the research group in strict accordance with the standard procedures. The operation is strictly carried out in accordance with the instrument and reagent instructions.

### 2.3. Observation Indicators

Use RA-800 to detect EFT and then measure the result of intrabatch precision. Taking the results of genetic testing as the gold standard, compare the sensitivity, specificity, and accuracy of EFT detection by scattering turbidimetry and direct colorimetry. The kappa test and ROC curve results of the diagnostic authenticity of the two methods were calculated.

### 2.4. Comparative Study of Clinical Performance Testing

#### 2.4.1. Repeatability

Choose one blood sample from normal population and one blood sample from thalassemia patients and use RA-800 to repeat the test of EFT 10 times each. Calculate the mean, standard deviation, and coefficient of variation, evaluate the precision within the batch, and then compare with the manufacturer's declared standard in the reagent manual.

#### 2.4.2. Method Comparison

From January 2021 to December 2021, a total of 100 cases of suspected thalassemia underwent prepregnancy physical examination at the Luohu District People's Hospital, of which 30 cases were genetically positive and 70 cases were negative. Use the EDTA anticoagulation vacuum blood collection tube to draw 2 mL of venous blood and store the specimen in the refrigerator at 2–8°C after receiving the specimen. Within 24 hours, the RA-800 and the KOFA detection system using the EFT detection kit were used for detection. The calculated hemolysis percentage value is compared with the reference interval of the two reagent instructions to judge the EFT test result. The clinical diagnosis based on genotype is the gold standard.

### 2.5. Statistical Analysis

Using SPSS 20.0 statistical analysis software, the measurement data conforming to the normal distribution are expressed as the mean ± standard deviation (*χ* ± *s*), and the comparison between the two groups uses the *t* test. Enumeration data are expressed as rate (%). The *χ*^2^ test was used for comparison between the two groups, and the difference was statistically significant at *P* < 0.05. The consistency checks use the kappa test.

## 3. Results

The precision comparison results of the kit used by RA-800 in the same batch are given in Table 1. The result meets the manufacturer's declaration standard in the reagent manual.

The results of the kappa test of diagnostic consistency using the two methods of RA-800 and KOFA are given in Table 2. RA-800 uses the scattering turbidimetric method, and KOFA uses the direct colorimetric method. The kappa value is 0.558, and the conclusion is that the consistency between the two is moderate.

With genetic diagnosis as the gold standard, the performance indicators of the two methods are given in Table 3. The scattering turbidimetry used by RA-800 is less sensitive, but its specificity and accuracy are higher than the direct colorimetry of KOFA.

The ROC curve drawn by the two methods is shown in Figure 1. The area under the ROC curve AUC of the two methods are equal, indicating that the authenticity and diagnostic value of the two methods are equal.

## 4. Discussion

Mature red blood cells are in the shape of double concave discs, and their surface area and volume are relatively large, which is conducive to gas exchange and self-deformation [11]. When red blood cells are in a hypotonic sodium chloride solution, they will swell rapidly until they are broken, causing changes in the intensity of scattered light [12, 13]. The rate of change of scattered light intensity per unit time is positively correlated with the percentage of red blood cell hemolysis, and the percentage of hemolysis can reflect the intensity of red blood cell osmotic fragility [14]. Increased osmotic fragility can be seen in hereditary spherocytosis, hereditary elliptic polycythemia, autoimmune hemolytic anemia, obstructive jaundice, and other diseases [15, 16]. The reduction can be seen in various types of globin genesis anemia, various hemoglobinopathies, iron deficiency anemia, and other diseases [17]. Therefore, the scope of its clinical application has been continuously expanded in recent years. There are many clinical methods to detect EFT, among which the single-tube method of red blood cell osmotic fragility detection is relatively simple. It is widely used in the initial screening of this disease in many areas with high incidence of thalassemia.

With the development of highly automated and informatized laboratories, most cumbersome methods have been gradually eliminated. At present, there are many fully automatic methods that are widely used in clinics, but the requirements for clinical laboratories are high, and the machines are expensive [18]. Moreover, these instruments are used for incidental detection of EFT, which has poor specificity and is not suitable for the preliminary screening of thalassemia in economically underdeveloped areas and grassroots hospitals.

The performance verification experiment in this study is to use KOFA by direct colorimetry and RA-800 by scattering turbidimetry to detect the EFT results of the blood samples of 100 subjects, respectively. Then, the methodological performance of the two methods is compared and analyzed. The results show that the sensitivity of RA-800's scattering turbidimetry is slightly lower than that of KOFA's direct colorimetry, but its specificity and accuracy are higher than that of KOFA. The kappa value of the diagnostic consistency test of the two methods is 0.558, and the conclusion is that the consistency of the two is moderate. The area under the ROC curve of the two is equal (AUC = 0.831), indicating that the diagnostic authenticity and diagnostic value of the two are equal. The above results indicate that the RA-800 performance index of the fully automatic red blood cell permeability fragility analysis using the scattering turbidimetry meets the clinical requirements. The sample can be tested without any processing of a separate machine, and there is no need to establish a laboratory pipeline, which can realize fully automated and lightweight testing EFT.

The current gold standard for clinical thalassemia detection is genetic diagnosis [7]. However, the test method is complicated, requires high technical and laboratory requirements, and is expensive. It is not suitable as a preliminary screening index for thalassemia screening. Therefore, it is difficult to screen for thalassemia in economically backward areas and basic hospitals and the community as a means of screening. In view of this study, some scholars proposed to use high specificity and high sensitivity indicators for detection to improve the positive and negative predictive values. This can make the test results more reliable and reduce the missed and misdiagnosed thalassemia.

## 5. Conclusion

The performance index of the new fully automatic red blood cell permeability fragility analyzer RA-800 meets the clinical requirements and has the advantages of simplicity, economy, and effectiveness. It is more suitable for economically backward areas, primary hospitals, and communities. The combination of RA-800 and blood analyzers for screening can effectively improve the positive and correct rate of thalassemia detection. It is particularly important for missed diagnosis, misdiagnosis, and genetic counseling for thalassemia.

## Figures and Tables

**Figure 1:** ROC curve for evaluating diagnostic tests.

**Table 1:** Comparison of hemolysis percentage of two blood specimen with manufacturer's standard accuracy.

Specimens	Repeat times (*n*)	Average hemolysis percentage (%)	Variation coefficient (%)	Vendor standard (%)	Result
Normal	10	77.0	2.2	≤6	Qualified
Thalassemia	10	55.0	3.7	≤6	Qualified

**Table 2:** Two methods of diagnosis consistency kappa test results.

	KOFA positive	KOFA negative	Kappa	Result
RA-800 positive	21	4	0.558	Moderate consistency
RA-800 negative	15	60		

**Table 3:** The coincidence of the two results with the genetic diagnosis results.

	Positive genetic diagnosis	Negative genetic diagnosis	Sensitivity (%)	Specificity (%)	Accuracy (%)
RA-800 positive	20	5	66.67	92.86	85.00
RA-800 negative	10	65			
KOFA positive	23	13	76.67	81.43	80.00
KOFA negative	7	57			

## Data Availability

The data used to support the findings of this study are available from the corresponding author upon request.
